# Planning and Design of a Full-Outer-Air-Intake Natural Air-Conditioning System for Medical Negative Pressure Isolation Wards

**DOI:** 10.1155/2021/8872167

**Published:** 2021-03-25

**Authors:** Chien-Lun Weng, Lih-Jen Kau

**Affiliations:** Department of Electronic Engineering, National Taipei University of Technology, No. 1 Sec. 3, Chung-Hsiao E. Rd., Taipei 10608, Taiwan

## Abstract

In the beginning of 2020, the coronavirus (COVID-19) pandemic started to spread globally, causing panic to the lives of people around the world; many countries executed lockdown of cities or even total lockdown of the entire countries. The coronavirus disease (COVID-19) is transmitted via air droplets. In medical environments that use traditional hermetic ventilation systems, medical personnel who come in contact with patients are more susceptible to infection compared to regular staff; therefore, the air flow and air quality of hermetic negative pressure isolation wards are highly critical. For this purpose, the study proposes a full-outer-air-intake natural air-conditioning system for negative pressure isolation wards. This innovative system draws in large amounts of fresh external air to greatly improve the air exchange rate in wards; negative pressure environments can be implemented depending on requirements to solve the issue of nosocomial infections in traditional negative pressure isolation wards that draw air from within the hospital. This greatly reduces the probability of nosocomial infection and infection via air droplets; furthermore, the system's intake and exhaust paths are completely isolated, solving the issue of air cross-contamination. Based on the results from the experiment site, this innovative system was designed and implemented based on the guidelines of hospital facilities and achieved air exchange per hour in excess of 12 times/hour, reaching a maximum of 54.5 times/hour. Indoor CO_2_ concentration was 576 ppm, negative pressure was −14 Pa, indoor temperature was 23.3°C, indoor humidity was 54.1%, and sensible heat exchange efficiency (*η*s) was 105.88% which effectively reduced ventilation load. Therefore, this innovative full-outer-air-intake natural air-conditioning system can provide medical staff and patients with a safe and healthy environment that prevents cross-infection.

## 1. Introduction

The coronavirus (COVID-19) pandemic spread globally, causing panic to the lives of people across the world. On March 11, 2020, the World Health Organization (WHO) announced that COVID-19 has become a global pandemic, which has infected over 7 million people and resulted in deaths of 430,000 people across 188 countries/regions [1]. This tragedy has not yet ceased and is instead continuing mercilessly, causing many countries to issue lockdown in cities and even total lockdown of the entire nations.  Figure 1 shows that the coronavirus (COVID-19) is transmitted via air droplets; therefore, there are several possible paths of transmission that can spread the virus between humans. Through coughing/sneezing, human carriers of the virus can atomize and produce virus-carrying droplets (particle size >5 *μ*m) and aerosols (particle size <5 *μ*m). The large droplets primarily float and settle in the air resulting in human infection; small aerosol particles are effectively dispersed in the air and can cause infection when inhaled into the human respiratory tract [2]. The virus can even be transmitted when people hold conversations [3–6]. Besides, human activity in enclosed spaces [7–9] is also one of the factors that has increased the infection rate of the coronavirus (COVID-19).

In the beginning of 2020, as many as 8000 medical personnel were infected in Italy, in which 63 physicians died from infection, resulting in a collapse of the frontline medical system. The primary factor was direct contact in enclosed medical environments between patients and medical staff, causing medical staff to be more prone to infection than general personnel. Another factor is the insufficient number of negative pressure isolation wards/spaces for admitting confirmed and suspected patients. The airflow, air quality, and pathogenic concentration are extremely relevant and important; plans for introducing fresh air to improve indoor air quality and airflow not only protect medical personnel but also, more importantly, prevent the problem of nosocomial infection [10].

Current negative pressure isolation wards contain ventilation systems that are generally well planned, but the issue of nosocomial and air cross-contamination is primarily due to the factor of indoor air quality (IAQ) and the airflow pathways of ventilation systems. When introducing external air, consideration must be given to the cleanliness and heat load of outside air; this is because the heat load of external air will increase ventilation system load and result in wasted resources and increased energy expenditure. Ventilation systems not only create safe and healthy indoor environments but also increase ventilation load, causing emissions that create heat and air pollution in the environment; this will bring about another unprecedented catastrophe due to environmental destruction.

### 1.1. Negative Pressure Isolation Ward Ventilation Systems' Overview

High-efficiency ventilation systems are a key element in medical environments. They stem heat load and pollutants from external environments while maintaining comfort and cleanliness within buildings; many utilize hermetic designs by planning ventilation systems in specific areas to maintain indoor air quality. To control the indoor air quality, the intake end of a ventilation system requires the installation of primary and intermediate filters; additionally, environment humidity must be controlled between 50 and 60%, and temperature must not fall below 22°C. The optimal temperature environment is 25°C∼27°C [11]. Negative pressure isolation wards are primarily for receiving patients with infectious disease to prevent transmission to medical personnel via air droplets, aerosols, or air carrying the virus to other areas through ventilation systems, causing nosocomial infections. The most common infection within a hospital is urinary tract infections, followed by respiratory tract infections [10].

### 1.2. Influencing Factors of Air Quality in Negative Pressure Isolation Wards

The factors that influence indoor air quality in medical spaces can generally be divided into 2 categories. The first is intrusion by external air pollution sources such as waste gas emissions from factories and traffic, particulate matter, ozone (O_3_), and other pollutant gases into rooms; the second category includes pollutant gases that are directly generated indoors, such as volatile organic compounds (VOCs) from indoor décor and carbon dioxide (CO_2_) exhaled by humans and microorganisms such as mould and bacteria [12].

Indoor air quality in medical spaces is a crucial factor of nosocomial infections; therefore, the impact on indoor air quality can be represented by the distribution of pollutant concentration. The concentration of indoor air pollutants can be explored from both pollutant generation and elimination aspects. In addition, CO_2_ concentration in indoor environments is a key indicator of indoor air quality; the indoor air quality of hospitals holds a CO_2_ concentration requirement of less than 600 ppm [13–15].

### 1.3. Improving Air Quality of Negative Pressure Isolation Wards via Full-Outer-Air-Intake

In recent years, much promotion has been given to the indoor air quality of buildings and the relationship with energy conservation. When a building's ventilation system is in operation, the indoor CO_2_ concentration settings can be controlled by CO_2_ sensors to maintain indoor air quality and reduce wasted energy [16, 17]. CO_2_ sensors can also be used to detect indoor CO_2_ concentration and thus build a CO_2_ concentration prediction model for the building to achieve more accurate control of indoor air quality as well as energy conservation [18–21]. Ventilation systems can be equipped with throttle valves to restrict the introduction of external air while achieving energy conservation [22].

Although current medical facilities have considered mechanical exhaust system designs, there is still the issue of nosocomial infections [23–25]. According to the World Health Organization (WHO), there are 14 cases of nosocomial infection in every 1000 days of hospitalization, reaching a rate of 1.4%. During the COVID-19 pandemic, airborne-based nosocomial infections became more severe; the first issue in solving nosocomial infections is to improve indoor air quality and eliminate the factors of air cross-infections.

The motive of this study is to find a comprehensive method to improve indoor air quality, diminish air cross-infections, enhance intake/exhaust energy conversion, and reduce ventilation system load. Meanwhile, this study aims to plan and design an innovative full-outer-air-intake natural air-conditioning system that is equipped with the function of filtering aerosols (PM_10_ and PM_2.5_) in the air for negative pressure isolation wards. By applying the system in negative pressure isolation wards, the primary purpose of this study is to introduce fresh external air, improve indoor air quality of wards, solve the issue of nosocomial infections, and provide medical personnel as well as patients with a safe space.

This article's structure is illustrated as follows: Section 2 details the structure of the innovative full-outer-air-intake natural air-conditioning system for negative pressure isolation wards; Section 3 details the actual case and experiment in this study; and Section 4 is the conclusion.

## 2. Structure of the Innovative Full-Outer-Air-Intake Natural Air-Conditioning System for Negative Pressure Isolation Wards

As mentioned above, this study aims to introduce fresh air to negative pressure isolation wards by creating a full-outer-air-intake natural air-conditioning system that provides a safe space for medical personnel and patients. Details of traditional ventilation systems in negative pressure isolation wards will be given to develop the structure of the full-outer-air-intake natural air-conditioning system; this section will provide details on system structure planning.

### 2.1. Structure of Traditional Ventilation Systems in Negative Pressure Isolation Wards

Negative pressure isolation wards refer to maintaining negative pressure up to 8∼12 Pa in the ward, hallways, or between wards, effectively preventing dirty air from entering other spaces through gaps as shown in Figure 2. Only when all of the openings (doors and windows) are closed between negative pressure isolation wards and hallways or nearby wards can the pressure difference be established effectively to prevent dirty air from leaking outside the ward. The internal and external pressure difference of the ward can be separated to *P*_1_ and *P*_2_; then, the pressure difference in the ward (Δ*P*) [26] is as shown in the following:

(1) $$\begin{array}{c} △P=P_{1}-P_{2}=\left(\xi_{1}+\xi_{2}\right)\frac{S^{2}\rho }{2}+H_{w}\left(P_{a}\right), \end{array}$$

where Δ*P* is the pressure difference; *H*_*w*_ is the friction drag, which is negligible as the gap depth of doors and windows is 10^−2^m; *ξ*_1_ is the local resistance that occurs when air enters from gaps in the walls and suddenly contracts the position. As the sectional area of the gap is very small, *ξ* approaches 0.5; *ξ*_2_ is the local resistance that occurs when air travels from the gaps of walls and suddenly expands the position. As the sectional area of the gap is very small, *ξ* approaches 1; *S* is the rate of airflow through the gap with the unit m/s; and *ρ* is the air density, which is approximately 1.2 kg/m^3^.

As shown in Figure 3, the current ventilation systems in negative pressure isolation wards utilize the method of greater air exhaust than air intake to create a negative pressure of at least 8∼12 Pa in an environment. The obvious difference in air pressure causes airflow to travel in a single direction from gaps in wards and hallway doors as well as the ability to withstand unavoidable differences in air pressure for short periods. This effectively expels air carrying virus from indoor spaces. Then, the air passes through a HEPA filter (high-efficiency particulate air filter) that catches viruses before being expelled outdoors [11]. The introduction of hospital air in the environment of negative pressure isolation wards can easily cause nosocomial infections via air cross-infections. From Figure 4, it is seen that when the negative pressure value of a ward is approximately 15 Pa, the opening of a door will cause the pressure difference to reduce to 0 Pa in 2 seconds, nearly balancing internal and external pressures. Therefore, when a door is opened, the airflow speed reflects the ability to prevent pollutants from entering; this has no correlation to the original pressure difference within the ward [27, 28].

The issue of nosocomial and air cross-infections exists in current negative pressure isolation wards; the primary influencing factor is due to the fact that the exhaust of current negative pressure isolation wards introduces hospital air, resulting in nosocomial air cross-infection instead of drawing in fresh external air. Providing a sufficient air exchange per hour can improve indoor air quality (IAQ), and another key factor is the issue of planning airflow pathways in ventilation systems. In addition, when the ward is opened, the pressure in the negative pressure ward will change rapidly, and such a rapidly changing pressure will be detected by the sensor. At this time, the exhaust air volume will be increased through the proposed exhaust system to avoid the air in the ward invading other areas.

### 2.2. Planning of the Innovative System Structure

The issue of nosocomial infections in current negative pressure isolation wards is primarily influenced by factors such as indoor air quality (IAQ) and the planning of airflow pathways in ventilation systems. This study utilized the properties of the full-outer-air-intake natural air-conditioning system in the general planning of ventilation systems for use in negative pressure isolation wards. By utilizing the building's internal and external steam partial pressure difference as the method of energy heat transfer, water was utilized to filter and purify air during heat exchange. This can capture particulate matters in the air while separating intake and exhaust pathways to comprehensively solve the issue of cross-contamination during air exchange [29]; when combined with the environmental controls of the ward, this can achieve minimum energy consumption and provide a safe space for medical personnel and patients.

During the planning of the full-outer-air-intake negative pressure isolation ward, introducing fresh external air into the ward to increase the air exchange per hour and to improve poor indoor air quality is a critically important influencing factor; first, one must understand the volume (*V*) of the negative pressure isolation ward as shown in the following:

(2) $$\begin{array}{c} V=W\times L\times H, \end{array}$$

where *V* is the volume of the ward with the unit of m^3^ and *W*, *L*, and *H* correspond to the width, the length, and the height of the ward, respectively, all with the unit of m.

In accordance with the Guidelines for Design and Construction of Hospitals [30] and the 2019 ASHRAE Handbook [28], the minimum standard for air exchange per hour must achieve 12 air exchanges, and the negative pressure difference of the ward must be a minimum of 8∼12 Pa; therefore, air exchange per hour and negative pressure difference are closely linked to fresh air intake and indoor exhaust. Air volume (*Q*) and air speed, as well as the sectional area of the intake/exhaust (*A*), are related as shown in (3) and (4). The air exchange per hour (*N*) of the negative pressure isolation ward is related to ward volume and intake/exhaust volume; air exchange per hour is related to diluting the virus concentration within the ward [31–35] as shown in (5) and shown in Table 1.

(3) $$\begin{array}{c} A=W\times L, \end{array}$$

where *A* is the area of the air vent with the unit of m^2^; *W* is the width of the air vent with the unit of m; and *L* is the length of the air vent with the unit of m.

(4) $$\begin{array}{c} Q=S\times A\times K, \end{array}$$

where *Q* is the air volume with the unit of m^3^/s; *S* is the air speed with the unit of m/s; *A* is the area of the air vent with the unit of m^2^; and *K* is the effective surface area factor, a constant number.

(5) $$\begin{array}{c} N=\frac{Q}{V}, \end{array}$$

where *N* is the air exchange per hour; *Q* is hourly air volume entering the ward represented with the unit m^3^/h; and *V* is the ward volume with the unit m^3^.

Based on the above assumption that air quality of the negative pressure isolation ward is related to air exchange per hour, we proposed a full-outer-air-intake natural air-conditioning system structure for the negative pressure isolation wards. We planned the completely separated intake/exhaust pathways for negative pressure isolation wards that are different from the planning of traditional ventilation systems as shown in Figure 3. In order to solve the issue of air cross-infections, air and water were used as carriers of energy conversion by using the building's steam partial pressure difference as the method of energy heat transfer; water can also filter and purify the air during heat exchange and capture all particulate matter in the air to provide negative pressure isolation wards with fresh air, improve indoor air quality, and effectively dilute virus concentration in the ward as shown in Figure 5.

### 2.3. Proposed Structure of the Innovative Environmental Control System

The planned operation structure of the indoor air quality and full-outer-air-intake natural air-conditioning system for negative pressure isolation wards can be separated into a sensing unit, set unit, central processing unit (CPU), and output control unit to the control system structure as shown in Figure 6. Different sensor components are used to collect environment data and set the target values of units to allow the CPU to calculate the required amount of fresh air needed by the negative pressure isolation ward to improve indoor air quality with minimum energy consumption and provide a safe medical space for medical personnel and patients.

Once the environmental control and function setting requirements of the negative pressure isolation ward are known, Figure 7 details the control structure of the full-outer-air-intake natural air-conditioning system. Planned items in the input end include temperature, humidity, indoor CO_2_ concentration, pressure, and ward volume; planned items for the output end include intake/exhaust air volume and air exchange per hour. Based on the temperature, humidity, pressure, and CO_2_ concentration data collected by the sensors, the CPU will calculate and determine the intake/exhaust air volume and air exchange per hour at the output end of the full-outer-air-intake natural air-conditioning system. The sensors will continue to collect and send data on the status of indoor air quality to adjust fresh air intake and exhaust air volume to maintain the air quality and pressure in the negative pressure isolation ward.

In this paper, we first explore the requirements of a negative pressure isolation ward with environmental factors such as indoor temperature, indoor humidity, heat load emitted from the human body, latent heat introduced from external air during exchange and sensible heat load, CO_2_ concentration, and negative pressure. All environmental factors can be detected using the environmental sensors of the sensing unit; detected environmental parameters are sent to the central processing unit, and during system operation, the CPU will also receive the set target ward bulk, negative pressure value, indoor temperature, and CO_2_ concentration signals. The CPU will perform neural network-like computing to obtain optimized intake air volume to maintain indoor air quality and comfort that achieves minimum energy consumption and maintains optimal operation efficiency for the full-outer-air-intake negative pressure natural air-conditioning system.

The control criterion of the proposed system is basically a kind of on/off control, but the control conditions are somewhat complicated. The main control parameters of the proposed system include indoor pressure, indoor CO_2_ concentration, and the number of air change rate (*N*). Once the door of the negative ward is opened and the negative pressure inside the ward is found to be insufficient, the exhaust air volume will be adjusted to the maximum to avoid the polluted air that may contain contaminants in the ward invading other areas. When the ward door is closed and the negative pressure value inside the ward is restored, the exhaust air volume will be reduced and operated with minimum air volume to maintain the negative pressure value in the ward. In addition, when the CO_2_ concentration in the ward exceeds 600 ppm, the air intake and exhaust volume will be increased so that the CO_2_ concentration in the ward can be reduced and be below 600 ppm. The above control criteria must comply with the requirement that the number of air change rate in the negative pressure ward shall not be less than 12 times per hour [28]. The control conditions of the proposed system are summarized as follows:

  Condition 1: when the pressure in the ward does not reach the minimum requirement of −12 Pa, the exhaust air volume of the system will be increased to prevent the air with pollutants in the ward from invading other areas
  Condition 2: when the pressure in the ward reaches the minimum requirement of −12 Pa, the exhaust system will maintain at an operation mode with minimum air volume
  Condition 3: when the CO_2_ concentration in the ward exceeds 600 ppm, the intake air volume and the exhaust air volume will be increased at the same time to introduce fresh air outside the hospital so that the CO_2_ concentration can be reduced
  Condition 4: when the CO_2_ concentration in the ward is lower than 600 ppm, the air intake and exhaust air volume will be maintained at an operation mode with minimum air volume
  Condition 5: when the number of air change rate in the ward is less than 12 times/hour, the frequency of the air intake and exhaust flow will be increased
  Note: the air-conditioning system in this test site is controlled by that of the medical institution

Negative pressure isolation wards must introduce fresh external air to improve indoor air quality; intake air volume must be greater than exhaust air volume to maintain negative pressure and simultaneously dilute virus concentration within the ward. Therefore, one must consider latent heat when introducing external air, sensible heat load, and the heat load emitted from human bodies when introducing fresh air. Total heat load is the primary factor that will affect the room's comfort level.

#### 2.3.1. Total Heat Load of the Human Body

Based on ASHRAE Standard 55a [36], heat generated from the human body (*Q*_*H*_) can be categorized as latent heat and sensible heat load; based on the number of patients in the ward (*n*), one can find total heat load of the human body as shown in (6)∼(8) [36].

The formula to calculate sensible heat from the human body is

(6) $$\begin{array}{c} Q_{Hs}=n\times \text{sensible heat load}. \end{array}$$

Human body's sensible heat load is 128.6 (W).

The formula to calculate latent heat load from the human body is

(7) $$\begin{array}{c} Q_{Hl}=n\times \text{latent heat load}. \end{array}$$

The human body's latent heat load is 58.1 (W).

The formula to calculate total heat load of the human body is

(8) $$\begin{array}{c} Q_{H}=Q_{Hs}+Q_{Hl}. \end{array}$$

#### 2.3.2. Latent Heat and Sensible Heat Load Introduced during Air Exchange

Based on the guidelines of ASHRAE Standard 62 [37], each member in a ward requires the amount of fresh air equal to 2.5 L/s; when air is exchanged in a room, external fresh air is introduced into the ward along with external heat. The heat load of external air can be categorized into sensible heat load and latent heat in calculations; the formula is shown in (9)∼(11) [37].

In this paper, *Q*_*O*_ is the outer air heat load, *V*_*p*_ is the ventilation rate, *Q*_*P*_ is the steam latent, *C*_*p*_ is the air specific heat capacity, Δ*T* is the internal/external temperature difference of the ward, and Δ*C* is the internal/external humidity difference of the ward.

The formula to calculate heat load of external air is

(9) $$\begin{array}{c} Q_{Os}=V_{p}\times C_{p}\times \Delta T. \end{array}$$

The formula to calculate latent heat load of external air is

(10) $$\begin{array}{c} Q_{Ol}=V_{p}\times Q_{p}\times \Delta C. \end{array}$$

The formula to calculate total heat load of external air is

(11) $$\begin{array}{c} Q_{O}=Q_{Os}+Q_{Ol}. \end{array}$$

The total heat load (*Q*_*T*_) of a negative pressure isolation ward primarily consists of the sum of the human body's heat load and external heat load introduced during air exchange; the formula for calculating total heat load of a ward is as follows:

(12) $$\begin{array}{c} Q_{T}=Q_{H}+Q_{O}. \end{array}$$

## 3. Experiment Configuration and Testing of the Full-Outer-Air-Intake Air-Conditioning System for Negative Pressure Isolation Wards

As mentioned above, the planning and design of the full-outer-air-intake natural air-conditioning system for negative pressure isolation wards proposed by this study was based on the Guidelines for Design and Construction of Hospitals [30] and ASHRAE. This section will provide details on the case planning of this study's full-outer-air-intake natural air-conditioning system for negative pressure isolation wards and conduct verification and description of performance.

### 3.1. Experiment Planning of the Full-Outer-Air-Intake Natural Air-Conditioning System for Negative Pressure Isolation Wards

The experiment site for this study was within the thoracic infection intensive care ward of a large hospital located in central Taiwan. Due to necessity from the COVID-19 pandemic, the thoracic infection intensive care ward was planned for repurposing as a negative pressure isolation ward. Each ward contained a room with a length of 3.7 m, width of 3.4 m, and height of 2.7 m for a ward volume of 33.97 m^3^; the experiment site is as shown in Figures 8–10 and based on the Guidelines for Design and Construction of Hospitals [30] and ASHRAE HVAC Applications [28]. As medical personnel must wear full personal protective equipment (PPE) including protective suits, goggles, and other relevant protective equipment when entering negative pressure isolation wards, indoor temperature shall be designed to be lower so that medical personnel and patients are comfortable; however, this temperature cannot fall below the baseline of 22°C. The CO_2_ concentration of indoor environments is a key indicator of indoor air quality and must be maintained below 600 ppm in medical environments; air exchange per hour is correlated with indoor CO_2_ concentration, and a minimum of 12 air exchanges per hour is required. The design conditions for the full-outer-air-intake natural air-conditioning system for negative pressure isolation wards are as shown in Table 2.

This study selected the full-outer-air-intake natural air-conditioning system, which uses the mass-energy conversion of air and water to exchange heat in the most natural method, as the primary ventilation system for negative pressure isolation wards. The energy conversion sensible heat efficiency (*η*s) can achieve 71∼112%. Airflow pathways are completely separated, solving the problem of air cross-contamination with the feature of creating positive or negative pressure environments based on design requirements [29]. The design is suitable for applications in the ventilation systems of negative pressure isolation wards. Design requirements are based on those in Table 2; the planning of the experiment site and equipment specifications used for the full-outer-air-intake natural air-conditioning system for negative pressure isolation wards are as shown in Table 3.

The system planning and configuration for the experiment site in this study is as shown in Figure 11. The ward exhaust was placed as close to the bed as possible to ensure that any viruses generated by the patient were removed from the room; exhaust length was 0.583 m, width was 0.38 m, and area was 0.2223 m^2^. Fresh air was introduced by the full-outer-air-intake natural air-conditioning system to maintain indoor air quality and reduce the amount of hospital air that enters the ward through gaps.

After the full-outer-air-intake natural air-conditioning system for negative pressure isolation wards was built, environment tests were conducted in the ward to evaluate critical performance indexes such as air exchange rate per hour, indoor temperature, indoor humidity, negative pressure, CO_2_ concentration, and sensible heat exchange efficiency according to the design specifications of Table 2. Equipment and specifications used for the evaluation are shown in Table 4. Based on ASHRAE 2000a [38], the measured results of outside air temperature (OA_*T*_), indoor air temperature (IA_*T*_), and intake air temperature (SA_*T*_) for the full-outer-air-intake natural air-conditioning system for negative pressure isolation wards were used to evaluate sensible heat exchange efficiency (*η*s) as in (13). The higher the sensible heat exchange efficiency, the lower the heat load of the incoming fresh air to the environment, which can effectively reduce the heat load of the air conditioner.

(13) $$\begin{array}{c} \eta_{S}=\frac{{\text{OA}}_{T}-{\text{SA}}_{T}}{{\text{OA}}_{T}-{\text{IA}}_{T}}\times 100\%. \end{array}$$

### 3.2. Performance Verification and Analysis

The full-outer-air-intake natural air-conditioning system for negative pressure isolation wards was built at the experiment site with the plans and design mentioned above. Once the system was built as shown in Figure 12, environmental tests were conducted in the ward to verify the operational benefits of the system. The key test indicator of negative pressure isolation wards is air exchange per hour which is correlated with indoor CO_2_ concentration; therefore, the test instrument Testo-480 was used to measure air speed at the exhaust. Equation (4) was used to calculate air volume; the area of the exhaust is 0.2223 m^2^, and air speed sample tests were performed at 8 points on the exhaust as shown in Figure 13. As the VAV fan of this innovative system is able to adjust air volume according to changes in the environment, samples were taken at the maximum air speed and minimum air speed; the air speed values at the 8 locations are as shown in Table 5. The average was taken as the air speed value of the exhaust: maximum average wind speed was 3.085 m/s, maximum exhaust air volume was 1,851.7 CMH, minimum average wind speed was 2.265 m/s, and minimum exhaust air volume was 1,359.5 CMH.

From Figure 14, the proposed innovative system for negative pressure isolation wards exhibited a maximum and minimum air exchange per hour of 54.5 and 40; both figures meet the minimum standard of 12 air exchanges per hour for negative pressure isolation wards. Air exchange per hour is closely correlated to indoor air quality and comfort. From Figure 15, it can be seen that temperature and humidity measured by the instrument TES-1364 showed indoor temperature at 23.3°C and indoor humidity at 54.1%; both figures meet the design requirements and medical environment guidelines of Table 1; when using the instrument MIC-98132S to measure CO_2_ concentration within the ward, indoor CO_2_ concentration was 576 ppm when 3 people were in the room, meaning CO_2_ concentration also cleared the design requirements and medical guideline CO_2_ concentration of 600 ppm. When this innovative system introduced fresh air, indoor air quality was maintained, and when the hermetic automatic doors of the ward closed, the negative pressure at the experiment site was −14 Pa as shown in Figure 16, meaning it effectively expelled and diluted harmful air in the ward to provide safe and good indoor air quality as well as a comfortable environment; when the hermetic automatic door opened, this system increased exhaust air volume due to the detection of insufficient pressure, and when the door was fully opened, negative pressure was 0 Pa. Maximum exhaust air volume was 1,851.7 CMH, ensuring that harmful gases invaded other nearby areas when the hermetic automatic door opened.

The full-outer-air-intake natural air-conditioning system for negative pressure isolation wards utilizes the steam partial pressure differences in the air and water evaporators to perform energy conversion and thus promoting indoor air exchanges.  Table 6 shows that outdoor air temperature (OA_*T*_) was 31.8°C, indoor air temperature (IA_*T*_) was 23.3°C, intake air temperature (SA_*T*_) was 22.8°C, and sensible heat exchange efficiency (*η*s) was 105.88%. When this system introduces fresh air into the ward, it effectively lowers the temperature of fresh outdoor air before allowing it indoors; through this system's energy conversion, condensation effects can capture outdoor microparticles before introducing cool, clean fresh air indoors to provide an environment of good air quality.

The feature of this innovative system utilizes air and water as energy carriers to use the difference of steam partial pressure in the air to perform energy conversion and achieve the effect of introducing outer air that is dehumidified and lowered in temperature and recover cold energy from the indoor exhaust; the intake and exhaust pathways are completely isolated, solving the problem of air cross-contamination. Therefore, this system is able to introduce mass amounts of fresh outer air to provide a high air exchange rate in wards; depending on environmental requirements, the system can also create negative environment pressure. This solves the problems of traditional negative pressure isolation wards which introduce air from within the hospital resulting in nosocomial infection. The system can effectively decrease the probability of infection via droplets and aerosols within the hospital to provide medical personnel and patients with good, safe air quality and a comfortable medical environment. This experimental site was originally a general intensive care unit of the infectious diseases department. Due to the COVID-19 epidemic, this ward was converted into a full-outer-air-intake negative pressure ward so as to provide treatment to confirmed patients. The overall project took 21 working days to complete the reconstruction. Compared with the construction of a new negative pressure ward, the construction time is greatly reduced. In addition to the application of the negative pressure isolation ward, the proposed innovative system can also be applied to other fields and environments, such as lecture halls and gymnasiums, to provide good indoor air quality.

In the traditional negative pressure ward, the ambient air inside the hospital is introduced, so it is easy to cause cross-infection problems in the hospital. Nevertheless, the proposed system introduces external air into the negative pressure ward, thus solving the major problem encountered in the traditional negative pressure ward. In addition, traditional hospitals use the outdoor air precooling air-conditioning system to introduce outdoor air, and since outdoor air is directly introduced, the heat load of the hospital's air conditioning is increased, thus leading to greatly increased air-conditioning energy consumption. Moreover, the fresh air introduced by the external air precooling air-conditioning system is directly supplied to the large area of the hospital, and not directly supplied to the negative pressure ward. The air in the negative pressure ward is introduced through door slits or other gaps, which can easily cause air infection problems in hospitals and fail to provide safe space for medical staff and patients.

Compared to the traditional system, the proposed system can introduce fresh outdoor air to provide a negative pressure ward with a maximum ventilation frequency of 54.4 times/hour, far exceeding the standard requirement of 12 times/hour. According to Table 1, when the number of air change rate exceeds 50 times/hour, it takes no more than 8 minutes to achieve a 99.9% removal rate of contaminants in the ward, which can effectively reduce the virus concentration and keep the CO_2_ concentration in the ward below 600 ppm. The proposed system not only has a high sensible heat exchange rate that effectively reduces the heat load of the air conditioning in the ward but also provides a healthy and safe medical environment. A comparison showing the superiorities of the proposed full-outer-air-intake air-conditioning system over traditional technologies can be found in Table 7.

As can be seen in Table 7, the proposed system can have a sensible heat exchange efficiency (*η*s) up to 105.88%. It is noted that a sensible heat exchange efficiency exceeding 100% means that the system has the effect of energy saving. Besides, the proposed system can reach an air change rate up to 54.4 times/hour, far exceeding 12 times/hour required by the specification, which shows the superiorities of the proposed system over traditional technologies.

## 4. Conclusion

In this paper, we have built a negative pressure ward that can be used for COVID-19 patients and successfully provided a safe medical space for medical staff and patients. In this paper, two commonly used indicators including sensible heat exchange efficiency (*η*s) and air change rate (*N*) are applied for performance evaluation. Based on the experimental results, the proposed innovative system can have an air change rate up to a range between 54.5 and 40 times/hour, which far exceeds the minimum requirement of 12 times/hour. The mass introduction of fresh air maintains indoor CO_2_ concentration below 600 ppm, achieving a CO_2_ concentration of 576 ppm, which also solves the problem of nosocomial infection encountered in most of the traditional negative pressure isolation wards. The proposed system also has isolated airflow pathways, comprehensively solving the issue of air cross-contamination that occurs during air exchange. In addition, the proposed system is capable of creating a negative pressure environment of −14 Pa depending on environmental requirements. Moreover, the proposed system utilizes air and water as energy carriers to use the difference of steam partial pressure in the air to perform energy conversion and achieve a sensible heat exchange efficiency (*η*s) of 105.88%, effectively reducing ventilation heat load. Negative pressure isolation wards are critical medical environments during the COVID-19 pandemic as they are the last line of defense for entire medical systems. Experiments have proved that the proposed system can be quickly deployed to various medical institutions, providing an energy-saving and safe medical environment for medical staff and patients.

## Figures and Tables

**Figure 1:** Transmission methods of COVID-19 [2].

**Figure 2:** Diagram of applying negative pressure to prevent the leak of harmful air.

**Figure 3:** Ventilation system diagram of current negative pressure isolation wards.

**Figure 4:** Changes in pressure difference during the process of door opening [27].

**Figure 5:** Structure diagram of the full-outer-air-intake natural air-conditioning system for negative pressure isolation wards.

**Figure 6:** Structure of the proposed full-outer-air-intake natural air-conditioning system for negative pressure isolation wards.

**Figure 7:** Control structure of the proposed full-outer-air-intake natural air-conditioning system for negative pressure isolation wards.

**Figure 8:** Experiment site of the proposed full-outer-air-intake natural air-conditioning system for negative pressure isolation wards.

**Figure 9:** Environment of experiment site-1.

**Figure 10:** Environment of experiment site-2.

**Figure 11:** Configuration of the proposed experiment site for the full-outer-air-intake natural air-conditioning system for negative pressure isolation wards.

**Figure 12:** Picture of the completed full-outer-air-intake natural air-conditioning system for negative pressure isolation wards.

**Figure 13:** Representation of air speed sample locations on the exhaust.

**Figure 14:** Diagram of air exchange per hour at the experiment site.

**Figure 15:** Indoor temperature, humidity, and CO_2_ concentration at the experiment site.

**Figure 16:** Negative pressure at the experiment site.

**Table 1:** Air exchange rate per hour (ACH) and the time (in minutes) required for airborne contaminants' removal with the efficiency of 90%, 99%, and 99.9%, respectively [35].

Air exchange rate per hour (*N*)	Minutes required for airborne contaminants' removal corresponding to different efficiencies		
	90%	99%	99.9%
1	138	276	414
2	69	138	207
3	46	92	138
4	35	69	104
5	28	55	83
6	23	46	69
7	20	39	59
8	17	35	52
9	15	31	46
10	14	28	41
11	13	25	38
12	12	23	35
13	11	21	32
14	10	20	30
15	9	18	28
16	9	17	26
17	8	16	24
18	8	15	23
19	7	15	22
20	7	14	21
25	6	11	17
30	5	9	14
35	4	8	12
40	3	7	10
45	3	6	9
50	3	6	8

**Table 2:** Design conditions of the full-outer-air-intake natural air-conditioning system for negative pressure isolation wards.

Item	Name	Data
1	Ward bulk (m^3^)	33.97
2	Indoor temp. (°C)	23∼25
3	RH (%)	50∼60
4	CO_2_ concentration (ppm)	600
5	Negative pressure (Pa)	8∼12
6	Air exchange per hour	12

**Table 3:** Equipment specifications of the full-outer-air-intake natural air-conditioning system.

Item	Name	Data
1	Size (*L* ∗ *W* ∗ *H*)	1,000 ∗ 930 ∗ 750 mm
2	Air volume (m^3^/h)	1,300∼1,800
3	Rated consumed power (W)	400
4	CO_2_ concentration (ppm)	600
5	Phase/voltage/frequency	1Ø/220 V/60 Hz
6	Sensible heat exchange efficiency (%)	85∼150

**Table 4:** Specification chart of measurement instruments.

Brand	Model	Detection range
Testo	Testo-480	Temperature: −20°C∼+70°C
		Humidity: 0∼100% RH
		Pressure: −100∼+100 hPa
		Atmospheric pressure: 700∼1100 hPa
		Wind speed: 0∼+20 m/s
TES	TES-1364	Temperature: −20°C∼+60°C
		Humidity: 10∼95% RH
MIC	MIC-98132S	CO_2_: 0∼9999 ppm

**Table 5:** Maximum/minimum wind speed and average wind speed values taken at each sampling point on the exhaust.

Sampling point	1	2	3	4	5	6	7	8	Average value
Maximum air speed (m/s)	4.69	4.83	2.95	3.17	2.1	2.7	2.2	2.04	3.085
Minimum air speed (m/s)	3.88	4.02	2.14	2.36	1.29	1.89	1.19	1.35	2.265

**Table 6:** Intake air temperature and indoor air temperature of the innovative system.

Item	Name	Data
1	Outdoor air temperature (°C)	31.8
2	Indoor air temperature (°C)	23.3
3	Intake air temperature (°C)	22.8

**Table 7:** Performance and function comparison of the proposed full-outer-air-intake negative pressure ward and that of traditional technology.

Item	Proposed full-outer-air-intake negative pressure ward	Traditional negative pressure ward
Introduce fresh outer air	Yes	No
Air cross-contamination	No	Yes
CO_2_ concentration control	Yes	No
Exhaust air volume control	Yes	No
Sensible heat exchange efficiency (*η*s)	105.88%	No
Air change rate (*N*)	Max. 54.4 times Min. 40 times	≧12 times

## Data Availability

The parameters and test data regarding this research are available at https://reurl.cc/4m4eDK.
